RETRACTED

# Constructing a Predictive Model of Depression in Chemotherapy Patients with Non-Hodgkin's Lymphoma to Improve Medical Staffs' Psychiatric Care

**DOI:** 10.1155/2021/9201235

**Published:** 2021-07-17

**Authors:** Cheng Hu, Qian Li, Ji Shou, Feng-xian Zhang, Xia Li, Min Wu, Meng-jing Xu, Li Xu

**Affiliations:** ^1^Quality Control Department, The Third Hospital of Quzhou, China; ^2^Psychiatry Department, The Third Hospital of Quzhou, China; ^3^Nursing Department, The Third Hospital of Quzhou, China; ^4^Rehabilitation Department, The Second Affiliated Hospital and Yuying Children's Hospital of Wenzhou Medical University, China

## Abstract

**Objectives:**

Depression is highly prevalent in non-Hodgkin's lymphoma (NHL) patients undergoing chemotherapy. The social stress associated with malignancy induces neurovascular pathology promoting clinical levels of depressive symptomatology. The purpose of this study was to establish an effective depressive symptomatology risk prediction model to those patients.

**Methods:**

This study included 238 NHL patients receiving chemotherapy, 80 of whom developed depressive symptomatology. Different types of variables (sociodemographic, medical, and psychosocial) were entered in the models. Three prediction models (support vector machine-recursive feature elimination model, random forest model, and nomogram prediction model based on logistic regression analysis) were compared in order to select the one with the best predictive power. The selected model was then evaluated using calibration plots, ROC curves, and *C*-index. The clinical utility of the nomogram was assessed by the decision curve analysis (DCA).

**Results:**

The nomogram prediction has the most efficient predictive ability when 10 predictors are included (AUC = 0.938). A nomogram prediction model was constructed based on the logistic regression analysis with the best predictive accuracy. Sex, age, medical insurance, marital status, education level, per capita monthly household income, pathological stage, SSRS, PSQI, and QLQ-C30 were included in the nomogram. The *C*-index was 0.944, the AUC value was 0.972, and the calibration curve also showed the good predictive ability of the nomogram. The DCA curve suggested that the nomogram had a strong clinical utility.

**Conclusions:**

We constructed a depressive symptomatology risk prediction model for NHL chemotherapy patients with good predictive power and clinical utility.

## 1. Introduction

Non-Hodgkin lymphoma (NHL) is a common hematological malignancy, originating from the lymphoid tissues. Chemotherapy is one of the common treatment options for non-Hodgkin lymphomas. However, chemotherapy is considered a stressor causing psychological problems in patients with NHL [1]. Compared with patients not receiving chemotherapy, patients receiving chemotherapy are more likely to experience depression [2]. Previous studies report that the incidence of depression among patients undergoing chemotherapy is 16.8-45% [1, 3, 4].

RETRACTED

As we all know, disease itself may also be a stressor for psychologic burden. And stress also associated with malignancy induces neurovascular pathology promoting depression [5]. Depression can not only reduce the quality of life of the patients but also increase the recurrence rate as well as the risk of death [5–7]. Therefore, exploring potential risk factors related to depression in NHL patients undergoing chemotherapy is important, to help in promoting mental health care.

Previous research points out that depression relates to physical conditions, diseases, sociodemographic characteristics, treatments, psychosocial factors, and so on [8]. Despite numerous research have identified many factors associated with depressive symptomatology in NHL patients undergoing chemotherapy, no systematic assessment aimed at predicting the risk of depressive symptomatology in NHL patients undergoing chemotherapy exists. Fortunately, studies have also pointed out that the nomogram can be used as a predictive tool to predict the risk of disease occurrence [9]. Psychological-based self-report tools, such as Hamilton Depression Scale (HAMD) [10], Depression Self-Rating Scale [11], and Beck Depression Scale [12], are often used in clinical practice to assess depressive symptomatology [13]. Therefore, we hypothesized that based on clinical and epidemiological characteristics as well as those scoring systems of depression, an effective prediction model could be developed in predicting the likelihood of depressive symptomatology for NHL patients.

This study is aimed at establishing a nomogram predictive model of depressive symptomatology in patients with NHL to improve medical staffs' psychiatric care. This model can provide information suitable for clinical decision-making, identification of individuals at high risk of depressive symptomatology. This research provides new ideas for improving the life quality of the NHL.

## 2. Materials and Methods

### 2.1. Patients

We conducted a cross-sectional study of patients diagnosed with NHL in The Third Hospital of Quzhou from December 2016 to June 2020. Combined with preoperative medical information, telephone questionnaire surveys and community follow-up were conducted. Community follow-up is a survey of patient information in the community where the patient lives in order to improve patient compliance with the survey. Informed consent was obtained from the patients before the start of the study. Participants were required to fill the questionnaire under the guidance of a designated researcher who had received psychology training to ensure they accurately understood the content of the questionnaire. The study was approved by the Institutional Ethics Review Board of The Third Hospital of Quzhou (approval no. 2016003), and all patients were Chinese residents. The inclusion criteria were as follows: non-Hodgkin's lymphoma was confirmed by pathological diagnosis, no history of tumor and treatment, no psychotropic medication was used during the study period, the patient had undergone chemotherapy, and the patient did not have any organ failure. The exclusion criteria were as follows: lack of compliance, declined to participate, tumors of uncertain origin, probable metastatic tumors (this is because the condition of patients with metastatic tumors is complex and easily misdiagnosed), and fever or infection of unknown origin.

RETRACTED

### 2.2. Diagnosis of Depressive Symptomatology

The 17-item HAMD (HAMD-17) was used to assess the severity of depressive symptomatology in non-Hodgkin's lymphoma. The score for each item was 0-4 or 0-2 (distinct/severe, doubtful/mild, absent, and obvious, respectively) [14]. The total score of HAMD-17 was 0 to 54. As previously described, a total score of HAMD − 17 ≥ 8 indicates depression and patients were assigned to the depression group [15, 16]. The internal consistency of HAMD-17 is 0.83, the interrater reliability is 0.97, and the test-retest reliability was 0.81 [17–19]. Therefore, the HAMD-17 score demonstrates good reproducibility and strong feasibility for follow-up investigations.

### 2.3. Demographic and Clinical Information

The patient's demographic information (medical insurance, home place, marital status, per capita monthly household income, doctor-patient communication frequency, age, gender, education level, income level, etc.) and clinical data (hypertension, diabetes, hypercholesterolemia, psychiatric history, family history of NHL, targeted drug, pathological stage, and palindromia) were obtained for the included patients. Relevant data were obtained from the NHL's medical records.

### 2.4. Data Collection and Psychological Status Assessment System

The Social Support Rate Scale (SSRS) was used to measure the dimensions of social support. The total score of SSRS ranges between 12 and 65 points (0-33 points, low social support; 33-45 points, medium social support; and 46-65 points, high level of social support) [20]. The test-retest reliability of SSRS is 0.89-0.94, and Cronbach's coefficient is 0.92 [21]. The anxiety state was measured using the 21-item Beck Anxiety Inventory (BAI). Each item's score ranges from 0 to 3, with a maximum score of 63, and the total BAI score of 45 points is considered as a diagnostic indicator of anxiety [22]. The internal consistency of the questionnaire is 0.92 [12]. The sleep state was measured using the Pittsburgh Sleep Quality Index (PSQI) [23], with a Cronbach's coefficient of 0.805 [24]. The PSQI score ranges from 0 to 21, with higher scores indicating poorer sleep quality. The Social Impact Scale was used for further evaluation, including the four dimensions of social exclusion, economic discrimination, inherent shame, and social isolation [25]. Using the four-level scoring method, the scale was divided into the total score of 4 dimensions. The higher the score, the greater the social impact that the individual perceives. Cronbach's coefficient is 0.85~0.90, and the correlation coefficient of each dimension is 0.28~0.66 [25].

RETRACTED

The European Organization for Research and Treatment Cancer Quality of Life Department C30 (EORTC QLQ C30) was used to determine the quality of life of NHL patients. The Chinese version of EORTC QLQ-C30 has a total of 30 items, which is divided into 15 areas, namely, 5 functional areas (physical, role, cognitive, emotional, and social function), 3 multi-item symptom areas (fatigue, pain, nausea, and vomiting), 1 general health status, and 6 single items (shortness of breath, insomnia, loss of appetite, constipation, diarrhea, and financial difficulties). The items on the scale 1 to 28 use a 4-level Likert scoring method. The 29th and 30th items are scored into 7 levels, from 1 to 7 points. The scale score ranges from 30 to 126 points. The higher the score, the worse the quality of life. The Chinese version of EORTCQLQ-C30 has good reliability and validity [26].

### 2.5. Statistical Analysis

The patients were randomly divided into the training and validation (7 : 3) groups. The training group was used for diagnosis and prognostic analysis. The validation group was used to validate the prediction model. All statistical analyses were performed in R software (version 3.5.3).

Support vector machines and random forest models are also becoming more widely used in biology [27–29]. The SVM-RFE algorithm may be superior to linear discriminant analysis and mean square error methods in selecting relevant features and removing redundant features, especially when the sample size is small [30]. The random forest model also has been shown to have better advantages on many datasets [31]. It is also able to handle data at high latitudes and can calculate the importance of each feature, and it can balance errors for unbalanced datasets. Therefore, randomForest was also used as an alternative model. Besides, to prevent overfitting of the clinical prediction model, all preset factors were incorporated into the LASSO analysis, dimensionality reduction was done, and suitable predictive factors were screened [32]. Multivariate logistic regression model was used to establish the predictive model. The nomogram included the most significant factors to predict the risk of depressive symptomatology in patients with NHL [28, 29, 33]. A calibration curve was used to evaluate the accuracy of the nomogram [34]. To further quantify the identification performance of the nomogram, the *C*-index was calculated and the ROC curve was plotted [35]. The AUC value was between 0.7 and 1, indicating that the model had a good prediction accuracy [36]. To improve medical staffs' psychiatric care (i.e., the ability to make better decisions using the model) by quantifying the net income under different threshold probabilities from patient's information, the DCA was used to evaluate the clinical applicability of the nomogram [9]. All statistical tests were two-sided, and *p* values less than 0.05 were considered statistically significant. This study proposed a visual multivariate prediction model to predict the incidence of depressive symptomatology in NHL patients [37].

RETRACTED

## 3. Results

### 3.1. Clinicopathological Characteristics

The recruitment process is illustrated in Figure 1. The clinical information of 238 NHL patients (140 males and 98 females) obtained between December 2016 and June 2020 was evaluated. The patients were divided into the depressive symptomatology group (80 patients) and nondepressed group (158 patients).  Table 1 shows the general characteristics of patient data. There were no significant differences between medical insurance, home place, doctor patient communication frequency, hypertension, diabetes, hypercholesterolemia, psychiatric history, family history of NHL, targeted drug, pathological stage, International Prognostic Index (IPI), palindromia, and the first time in hospital in NHL patients with and without depressive symptomatology. There were statistically significant differences between age, gender, education level, marital status, per capita monthly household income, disclosure of NHL diagnosis, SSRS, BAI, PSQI, and Social Impact Scale in the two groups.

### 3.2. Prediction Model Selection and Screening Predictors

The flow chart of model screening and evaluation design is illustrated in Figure 2(a). There were 167 cases in the training group and 71 cases in the validation group. The support vector machine-recursive feature elimination (SVM-RFE) was used to build a prediction model which may be better than linear discriminant analysis in selecting correlated features and removing redundant features. The SVM-RFE model had the highest accuracy (AUC = 0.8722) when it included 7 predictive factors (Figure 2(b)). The order of features in SVM-RFE method was ranked in Supplementary Table 1. In addition, randomForest forest models were also constructed to assess predictive ability (Figure 2(c)). Importance values of each factor in the random forest model were showed. And the ROC curve (AUC = 0.87) demonstrated the accuracy of the random forest model. We believe that the model can be further optimized. Overfitting of models is a challenge in machine learning. Therefore, we used the minimum absolute contraction selection operator (LASSO) method to further reduce the number of features to prevent overfitting of the prediction model. In this study, we randomly performed 1000 LASSO regressions and obtained the best combination of predictors. The predictors were then sequentially included in the logistic model based on the number of occurrences of the predictors. It was found that the model must have the most efficient predictive ability when 10 predictors are included (AUC = 0.938) (Figure 2(d)). In summary, we find that the model based on LASSO analysis combined with logistic regression has the strongest predictive power.

RETRACTED

Therefore, the LASSO regression model (Supplementary Figures 1(A) and 1(B)) was used to reduce the factors in this study from 24 predictors to 10 predictive parameters, thereby establishing a predictive model containing 10 predictors. The 10 predictive factors included education level, sex, age, marital status, medical insurance, per capita monthly household income, pathological stage, SSRS, PSQI, and QLQ-C30. Principal component analysis (PCA) revealed that these predictors could potentially distinguish between the depressed and nondepressed groups (Supplementary Figure 1(C)).

### 3.3. Establishment of the Prediction Model

The logistic model was used to analyze and determine the 10 predictive factors, and the nomogram is constructed in R software as shown in Figure 3. Among them, sex, age, education level, PSQI, and QLQ-C30 were found to be the most significant factors associated with the occurrence of depressive symptomatology in patients with NHL (*p* < 0.05). The specific performance of various factors in the prediction model of depressive symptomatology in patients with NHL is shown in Table 2.

### 3.4. Validation of the Prediction Model

The calibration curve of the nomogram showed good agreement between the observation and prediction (Figure 4(a)), indicating that the model can be used to assess the risk of depressive symptomatology in NHL patients. Besides, the AUC in the training group of the prediction model was 0.972, and the AUC in the verification group was 0.856 (Figure 4(b)). The *C*-index in the overall sample and verification group indicated the good predictive performance of the nomogram (the *C*-index of the overall sample was 0.944, and the *C*-index of the verification group was 0.885) (Table 3).

RETRACTED

### 3.5. Evaluation of Clinical Application

The decision curve analysis (DCA) of the nomogram is shown in Supplementary Figure 2. The results show that the decision curve based on the nomogram predictive model can help in making better clinical decisions. This means that the established predictive model can improve medical staffs' psychiatric care, promote early planning of a clinical intervention, and better predict the risk of disease, hence support individualized intervention.

## 4. Discussion

Nomograms are widely used for prognostic predictive analysis in cancer prognosis, due to their ability to comprehensively integrate risk factors in multiple dimensions. Besides, the logistic regression analysis results can be graphed and visualized, and this greatly improves the accuracy of the predictions, which can be easily interpreted, hence suitable in clinical decision-making [38]. Obviously, there is no research on the application of a nomogram model to predict the risk of depressive symptomatology in NHL patients undergoing chemotherapy. Based on a total of 10 predictive factors, including the patients' general clinical data and evaluation of various dimensions of the quality of life, this study for the first time established and verified a nomogram prediction model as a predictive tool for depressive symptomatology in non-Hodgkin's lymphoma patients.

LASSO regression model was used in this study to screen and predict related factors and reduced the main factors from 24 to 10, and the factors included sex, age, education level, marital status, medical insurance, per capita monthly household income, pathological stage, SSRS, PSQI, and QLQ-C30. Based on the predicted factors, a nomogram prediction model containing 10 optimal features was established as a predictive tool for the occurrence of depressive symptomatology in non-Hodgkin's lymphoma patients. Similar to previous studies, most of these variables have been reported to be related to the occurrence of depression [39]. Internal validation of the nomogram using the validation cohort showed that the prediction tool had a good predictive ability. Therefore, the nomogram can help in the early prediction of non-Hodgkin's lymphoma patients with a high risk of depressive symptomatology and provide targeted medical care to improve the prognosis of patients.

RETRACTED

This study suggests that the risk factors for depressive symptomatology in patients with NHL undergoing chemotherapy include female, elderly, low education level, good marital status, medical insurance, high household income, lower pathological stage, SSRS, PSQI, and QLQ-C30. Numerous previous studies have reported that these factors are associated with a higher risk of depressive symptomatology in patients with lymphoma, similar to the results of previous systematic reviews [8]. Polikandrioti et al. pointed out that the elderly group has a higher risk of depressive symptomatology compared to the younger population [40]. Four studies with 1,149 participants reported that female participants had a higher risk of depressive symptomatology compared to male participants [1, 3, 41, 42]. Good marital status also helps to prevent depressive symptomatology. Previous research reports that reduced sex life is significantly related to depression in cancer patients undergoing chemotherapy [43]. The type of medical insurance is also an important factor influencing depression in patients with NHL. This study showed that patients using agricultural insurance and self-financed payment methods were at a higher risk of developing depressive symptomatology. Anticancer treatment is expensive, and the economic burden placed on the patients has a greater negative impact on the patients' emotional and mental health [44]. Research reports that patients with higher cancer stages are at higher risk of depressive symptomatology [3, 45–48]. Numerous studies have reported that sleep disorders are positively related to increased risk of depressive symptomatology [49–51]. Two studies, with 366 participants, provided evidence that patients with sleep disorders had higher depression scores than those with no sleep disorders [50, 51]. Consistent with previous studies, this study found that lack of social support was significantly associated with depression [52, 53]. Depression can be prevented through good social relationships, which can buffer against stressful environments [54]. Depression also restricts social interaction activities, leading to a decline in the quality of life. Studies have reported that the self-evaluation of cancer patients can greatly affect the patient's mental health and disease prognosis [9]. Self-evaluation is likely to affect how people feel, think, and act, and also affect their assessment of stress stimuli [55].

Therefore, medical workers should take some preventive measures to improve psychiatric care for patients at high risk for depressive symptomatology. Psychological interventions for such patients should be strengthened to ease their negative emotions, strengthen their awareness of the disease and treatment, and enhance their confidence in overcoming the disease, hence face life and the disease with a more positive and optimistic attitude [8, 56]. Besides, the patients' relatives and friends should play an active role in providing social support to the patients, which further improves their psychological conditions. At the same time, the psychological condition of the patients should be regularly monitored for prevention and early diagnosis of depressive symptomatology.

RETRACTED

The proposed nomogram is innovative in the following aspects. Firstly and most importantly, this was the first prognostic nomogram established for patients with non-Hodgkin's lymphoma, making individualized screening possible. Secondly, as the new net benefit analysis method, DCA analysis was applied to our nomogram, and the results showed that the model had a good clinical application value. Finally, early intervention can reduce the risk of depressive symptomatology in NHL patients. The significance of the findings was encouraging, and the predictive model has satisfactory clinical utility. However, some potential limitations should be considered. And the predictive model requires further external validation and multicenter studies to confirm its clinical applicability. Besides, it also remains unknown if the model is acceptable by medical workers and patients.

In this study, we established and validated a nomogram for predicting the risk of depressive symptomatology in patients with NHL undergoing chemotherapy. Our study also found that risk factors for depressive symptomatology in NHL patients receiving chemotherapy included the following: female, elderly, low education level, good marital status, medical insurance, high household income, lower pathological stage, SSRS, PSQI, and QLQ-C30. The significance of the findings was encouraging, and the predictive model has satisfactory clinical utility.

By using this predictive model, individuals at high risk for NHL can be identified prior to clinical manifestation. Medical staffs could take some preventive measures for high-risk depressive symptomatology at early time. Psychological interventions for such patients should be strengthened to ease their negative emotions, strengthen their awareness of the disease and treatment, and enhance their confidence in overcoming the disease, hence face life and the disease with a more positive and optimistic attitude. Therefore, early intervention can reduce the risk of depressive symptomatology in patients with NHL, reduce the consumption of precious medical resources, facilitate further clinical research, and provide personalized care plans to improve quality of life.

RETRACTED

## 5. Conclusion

In conclusion, we established and validated a nomogram for predicting the risk of depressive symptomatology in patients with NHL undergoing chemotherapy. The proposed nomogram showed relatively high accuracy. The model can help doctors and medical staff to determine the risk of depressive symptomatology in patients with NHL, and provide individualized care to improve the quality of life of the patients.

## Figures and Tables

**Figure 1:** Flow chart of the study design.

**Figure 2:** Prediction model selection. (a) Flow chart of model screening and evaluation design. (b) The support vector machine-recursive feature elimination (SVM-RFE) was used to build a prediction model. The SVM-RFE model had the highest accuracy (AUC = 0.8722) when it included 7 predictive factors. (c) Importance values of each factor in the random forest model (the picture above). And the ROC curve (AUC = 0.87) demonstrated the accuracy of the random forest model (the picture below). (d) Based on the number of occurrences of each factor, it is incorporated into the logic model to obtain a pattern diagram of the AUC values (the picture above). Ultimately, the simplest predictive model with good predictive power can be constructed using only 10 predictors (the picture below).

**Figure 3:** Establishing a predictive model. The predictive model of depressive symptomatology in patients with NHL. Sex, age, medical insurance, marital status, education level, per capita monthly household income, pathological stage, SSRS, PSQI, and QLQ-C30 are significant factors affecting the occurrence of depressive symptomatology in patients with NHL (*p* < 0.05).

**Figure 4:** Validation of the prediction model. (a) Calibration curve of the prediction model of depressive symptomatology in patients with NHL (*B* = 10000). The *x*-axis is the predicted risk of depressive symptomatology in patients with non-Hodgkin's lymphoma. The *y*-axis represents the actual incidence of depressive symptomatology in patients with non-Hodgkin's lymphoma. The solid line represents the actual prediction of the prediction model. The more consistent the solid line and the dotted line are, the better the predictive ability of the predictive model. (b) AUC represents the accurate prediction of the risk of depressive symptomatology in patients with NHL in randomly selected cases. The AUC values of the training set (red) and validation set (blue) are 0.972 and 0.856, respectively.

**Table 1:** Patient characteristics.

Variables	Depressive symptomatology (*n* = 80)	No depressive symptomatology (*n* = 158)	*p* value
Age	57.4 ± 9.7	53.7 ± 14.5	0.041^∗^
Gender			*p* ≤ 0.001^∗∗^
Male	12 (15)	128 (81)	
Female	68 (85)	30 (19)	
Education level			*p* ≤ 0.001^∗∗^
Primary school or below	49 (61.2)	58 (36.7)	
Junior high school	21 (26.3)	61 (38.6)	
Senior high school or higher	10 (12.5)	39 (24.7)	
Marital status			0.014^∗^
Single	1 (1.3)	9 (5.7)	
Married	70 (87.4)	144 (91.1)	
Divorce	9 (11.3)	5 (3.2)	
Medical insurance			0.059
Self-paying	11 (13.8)	17 (10.8)	
Social security payments	57 (71.2)	105 (66.4)	
Commercial insurance payment	12 (15)	36 (22.8)	
Home place			0.32
Rural areas	33 (41.3)	57 (36.1)	
Urban areas	47 (58.7)	101 (63.9)	
Per capita monthly household income			0.027^∗^
≤4000 yuan/month	13 (16.3)	16 (10.1)	
400-8000 yuan/month	37 (46.3)	51 (32.3)	
>8000 yuan/month	30 (37.4)	91 (57.6)	
Doctor patient communication frequency			0.197
Less	15 (18.8)	43 (27.2)	
Normal	59 (73.7)	98 (62)	
Frequent	6 (7.5)	17 (10.8)	
Hypertension			0.788
No	63 (78.7)	122 (77.2)	
Yes	17 (21.3)	36 (22.8)	
Diabetes			0.977
No	73 (91.2)	144 (91.1)	
Yes	7 (8.8)	14 (8.9)	
Hypercholesterolemia			0.549
No	64 (80)	121 (76.6)	
Yes	16 (20)	37 (23.4)	
Psychiatric history			0.599
No	77 (96.2)	155 (98.1)	
Yes	3 (3.8)	3 (1.9)	
Family history of NHL			0.544
No	75 (93.7)	152 (96.2)	
Yes	5 (6.3)	6 (3.8)	
Targeted drug			0.334
No	60 (75)	109 (69)	
Yes	20 (25)	49 (31)	
Pathological stage			0.372
No	31 (38.7)	52 (32.9)	
Yes	49 (61.3)	106 (67.1)	
IPI			0.067
Score 0 to 2	28 (35)	75 (47.5)	
Score 3 to 5	52 (65)	83 (52.5)	
Palindromia			0.791
No	19 (23.8)	40 (25.3)	
Yes	61 (76.2)	118 (74.7)	
The first time in hospital			0.874
No	22 (27.5)	45 (28.5)	
Yes	58 (72.5)	113 (71.5)	
Disclosure of NHL diagnosis			*p* ≤ 0.001^∗∗^
No	7 (8.8)	58 (36.7)	
Yes	73 (91.2)	100 (63.3)	
SSRS			*p* ≤ 0.001^∗∗^
Low	20 (25)	57 (36)	
Medium	42 (52.5)	96 (60.8)	
High	18 (22.5)	5 (3.2)	
BAI			*p* ≤ 0.001^∗∗^
Negative	30 (37.5)	112 (70.9)	
Positive	50 (62.5)	46 (29.1)	
PSQI	9.3 ± 2.3	4.8 ± 3.3	*p* ≤ 0.001^∗∗^
Social Impact Scale	60.1 ± 8.1	62.6 ± 7.6	0.017^∗^
Total score QLQ-C30	51.7 ± 8.8	59 ± 12	*p* ≤ 0.001^∗∗^

^∗^ *p* < 0.05 and ^∗∗^*p* < 0.01. Values are presented as the mean ± SD or number (percent (%)). IPI: International Prognostic Index; SSRS: Social Support Rate Scale; BAI: Beck Anxiety Inventory; PSQI: Pittsburgh Sleep Quality Index.

RETRACTED

**Table 2:** Prediction factors for depressive symptomatology.

Variable	Prediction model		
	*β*	Odds ratio (95% CI)	*p* value
(Intercept)	1.744	5.719 (0.108-315.986)	0.390
Sex	4.348	77.361 (24.273-313.424)	*p* ≤ 0.001
Age	0.056	1.058 (1.015-1.106)	0.011
Education_level	-0.833	0.435 (0.214-0.84)	0.016
Marital_status	0.136	1.145 (0.207-6.633)	0.878
Medical_insurance	-0.460	0.631 (0.276-1.416)	0.266
Per_capita_monthly_household_income	0.310	1.364 (0.726-2.61)	0.338
Pathological_stage	-0.311	0.733 (0.279-1.908)	0.523
SSRS	-0.335	0.715 (0.339-1.492)	0.373
PSQI	0.170	1.185 (1.023-1.387)	0.027
Total_score_QLQ_C30	-0.144	0.866 (0.808-0.918)	*p* ≤ 0.001

*β* is the regression coefficient.

**Table 3:** *C*-index of the prediction model.

Dataset group	*C*-index of the prediction model	
	*C*-index	The *C*-index (95% CI)
Training set	0.972	0.938-1.000
Validation set	0.885	0.796-0.974
Entire cohort	0.944	0.907-0.981

## Data Availability

The datasets generated and analyzed during the present study are available from the corresponding author on reasonable request.

## Abbreviations

BAI: Beck Anxiety Inventory
DCA: Decision curve analyses
HAMD-17: The 17-item HAMD
IPI: International Prognostic Index
LASSO: Least absolute shrinkage and selection operator
NHL: Non-Hodgkin's lymphoma
PCA: Principal component analysis
PSQI: Pittsburgh Sleep Quality Index
QLQ-C30: European Organization for Research and Treatment Cancer Quality of Life Department C30
ROC: The receiver operating characteristic curve
SIS: Social Impact Scale
SVM-RFE: Support vector machine-recursive feature elimination
SSRS: Social Support Rate Scale

## Supplementary Materials

Supplementary Materials This section contains the raw data from all patients participated in the study.
